# Small Extracellular Vesicles: A Novel Avenue for Cancer Management

**DOI:** 10.3389/fonc.2021.638357

**Published:** 2021-03-15

**Authors:** Yanan Gao, You Qin, Chao Wan, Yajie Sun, Jingshu Meng, Jing Huang, Yan Hu, Honglin Jin, Kunyu Yang

**Affiliations:** Cancer Center, Union Hospital, Tongji Medical College, Huazhong University of Science and Technology, Wuhan, China

**Keywords:** small extracellular vesicles, exosomes, early cancer detection, drug delivery systems, therapeutic strategy

## Abstract

Extracellular vesicles are small membrane particles derived from various cell types. EVs are broadly classified as ectosomes or small extracellular vesicles, depending on their biogenesis and cargoes. Numerous studies have shown that EVs regulate multiple physiological and pathophysiological processes. The roles of small extracellular vesicles in cancer growth and metastasis remain to be fully elucidated. As endogenous products, small extracellular vesicles are an ideal drug delivery platform for anticancer agents. However, several aspects of small extracellular vesicle biology remain unclear, hindering the clinical implementation of small extracellular vesicles as biomarkers or anticancer agents. In this review, we summarize the utility of cancer-related small extracellular vesicles as biomarkers to detect early-stage cancers and predict treatment outcomes. We also review findings from preclinical and clinical studies of small extracellular vesicle-based cancer therapies and summarize interventional clinical trials registered in the United States Food and Drug Administration and the Chinese Clinical Trials Registry. Finally, we discuss the main challenges limiting the clinical implementation of small extracellular vesicles and recommend possible approaches to address these challenges.

## Introduction

Extracellular vesicles (EVs) are small lipid bilayer-bound vesicles released from living cells into the extracellular environment. These vesicles lack functional nuclei and cannot replicate (1). Traditionally, EVs can be roughly classified into two main subtypes regarding their characteristics and biogenesis pathway: ectosomes and small extracellular vesicles (sEVs). Ectosomes have a diameter between 100 and 1000 nm and are generated by cytoplasmic membrane budding (2). sEVs, also referred to as “exosomes” by some researchers, are smaller in diameter (30–150 nm) and released by the fusion of the multivesicular bodies (MVBs) with the plasma membrane. According to the updated guidelines of the International Society for Extracellular Vesicles of 2018 (MISEV2018), when naming a new EV subtype, the term “EVs” is recommended, followed by a description of vesicle features, such as size, density, cell of origin, and experimental conditions, making EV names more descriptive and informative (2, 3). Some experts have a greater attachment to the traditional term “exosomes” and we consider it quite a personal preference to call them either “exosomes” or “small extracellular vesicles (sEVs)” (3). In congruence with the latest suggestion, we refer to “exosomes” as “sEVs” throughout this review.

In 2018, Zhang et al. discovered another group of non-membranous secretory extracellular nanoparticles (<50 nm) termed “exomeres”, which were initially identified by asymmetric flow field-flow fractionation (AF4) and consisted of various biological molecules (4). Later on, a simple ultracentrifugation-based method was employed to isolate exomeres from sEVs (5). Although the research on exomeres is limited by technical barriers, such as the rarity of AF4 and the lack of the universally recognized nomenclature system, researchers have reported some biological functions of exomeres. For example, the β-galactoside α2,6-sialyltransferase 1 (ST6Gal-I), an exomere protein from human colorectal cancer cells, could sialylate the β1-integrin of recipient cells. Another exomere protein amphiregulin (AREG) could serve as the EGFR ligand, regulate the EGFR signaling pathway in normal intestinal organoids, and significantly promote the growth of colonic cancer organoids (5). Although exomeres and sEVs have comparable protein profiles, the stability in the circulatory system regarding the absence of bilayered membrane, and the biological safety of exomeres *in vivo* are still unclear. However, similar issues related to sEVs have been well addressed with extensive investigation, leaving sEVs much more accessible therapeutic tools.

EVs play a critical role in intracellular hemostasis and intercellular communication. In 1946, researchers discovered that ultracentrifugation pellets of plasma could activate platelets and blood clotting factors; these effects were attributed to the EVs in the pellets (6, 7). Subsequently, reticulocyte-derived EVs were identified by electronic microscopy as “discarded waste” that maintains intracellular homeostasis during erythrocyte maturation (8, 9). As the knowledge of sEVs has grown exponentially since 2000, some research groups have unveiled more biological functions and established novel clinical applications of sEVs, especially sEVs as messengers in various pathological processes and an efficient and targeted drug delivery system (10–13). In this review article, we focus on the recent development of sEVs as biomarkers for early cancer detection and follow-up care, as well as therapeutic particles for cancer treatment.

## Small Extracellular Vesicles Biogenesis, Cargo Sorting, And Contents

sEV biogenesis is complex and involves the formation of specialized intracellular compartments, known as MVBs/late endosomes, a key sorting point in the endocytic pathway (14). The inward budding of MVB membrane produces numerous intraluminal vesicles (ILVs), a group of small (~25–30 nm in diameter) spheroids containing cytosolic components and certain proteins from the invaginated MVB membrane (15). ILVs are expelled into the extracellular environment when MVBs fuse with the plasma membrane, referred to as sEVs. sEVs are spheroids in solution but sometimes they display a sauce-like shape under transmission electron microscopy as an artifact of drying during preparation (16). Typically, sEVs collected by fraction collection have a density range from 1.1 to 1.2 g/ml (17). Alternatively, MVBs with ILVs can fuse with lysosomes for hydrolysis of endocytosed macromolecules (18). However, some ILVs can fuse with MVB membrane and the proteins of ILVs membrane can be incorporated into endosome or lysosome membrane, a process called “backfusion”. As a result, some ILV membrane proteins, such as tetraspanin proteins and mannose-6-phosphate receptors, can escape the lysosomal degradation and recycle to the trans-Golgi network or plasma membrane (15, 19) (**Figure 1**).

**Figure 1:** sEV biogenesis, cargo contents and uptake. HSP, Heat shock proteins; SCAMPs, Secretory carrier membrane proteins; ALIX, Apoptosis-linked gene 2–interacting protein X; HRS, Hepatocyte growth factor-regulated tyrosine kinase substrate; TSG101, Tumor susceptibility gene 101.

Although the formation of ILVs and the protein cargo sorting system have not been fully elucidated, researchers showed that the endosomal sorting complex required for transport (ESCRT) functions in this process (20). As complicated protein machinery, ESCRT consists of four main complexes (ESCRT-0, -I, -II, and -III) and works cooperatively with associated proteins (VPS4, VTA1, ALIX) to promote MVB and ILV biogenesis. The ESCRT-0 complex recognizes and sequesters ubiquitinated domains of endosomal membrane proteins *via* its ubiquitin-binding subunits, such as hepatocyte growth factor-regulated tyrosine kinase substrate protein (HRS); whereas ESCRT-I and-II facilitate the formation of the buds with sequestered proteins. Then the whole complex interacts with ESCRT-III/Vps4 complex, which stabilizes tubular endosomes and cleaves the bud to form ILVs (20, 21). Finally, the disassembly and recycling of ESCRT machinery requires the energy supplied by AAA-ATPase Vps4 (20). Besides, several ESCRT components (TSG101, ALIX) and ubiquitinated proteins have been identified in purified sEVs from various cell types. Typically, the sEV marker protein ALIX was reported to collaborate with other ESCRT proteins (TSG101 and CHMP4) and facilitate cargo selection, endosomal membrane budding and vesicle detachment in the form of syntenin-syndecan-ALIX complex (22). These results support the theory that ESCRT is critical in sEV biogenesis. However, some research indicated ESCRT-independent mechanisms for ILVs formation and release (**Figure 1**). Trajkovic et al. reported that the depletion of sphingomyelinases, instead of ESCRT inhibition, in oligodendroglial cells could significantly reduce the formation of MVBs and associated proteolipid protein (PLP)-enriched sEVs, an inspirational phenomenon referred to as “ceramide-dependent sEV biogenesis” (23). Further investigation showed that some lipid raft-based microdomains of the endosomal membrane contain numerous sphingomyelinases, enzymes hydrolyzing sphingomyelins to ceramides (24). Ceramides could induce negative curvatures of the endosomal membrane and lateral phase separation, thus functioning as coalescers in the process of ILV abscission (25, 26). Nonetheless, whether this ceramide-dependent machinery could be generalizable to other cell types and intraluminal contents is still unclear. Interestingly, some tetraspanins, such as CD63, CD82 and Tspan8, have been regarded as key points in cargo sequestration and sEVs formation, in a ceramide-independent and ESCRT-independent manner. Niel et al. reported that a CD63-dependent mechanism facilitated the formation and release of melanosomes-enriched sEVs, while downregulating CD63 led these melanosomes into ESCRT-dependent degradation in human melanoma cells (27). Similarly, the elevated expression of CD9 and CD82 could increase the secretion of β-catenin-enriched sEVs from human embryonic kidney 293 cells (HEK293), and a study utilizing the rat adenocarcinoma model showed that Tspan8 participated in the selective recruitment of proteins into sEVs (28, 29). Additionally, thousands of molecules have been reported to contribute to selective cargo sorting into ILVs and the release of sEVs, such as Rab GTPase (30), glycosphingolipids and flotillins (31), chaperone HSC70 (32, 33) and small integral membrane proteins of the lysosome/late endosome (SIMPLE) (34).

Similar to the specific recruitment of protein contents, the sorting of particular nucleic acids is dedicatedly monitored by multiple mechanisms. Generally, smaller size, higher abundance, and greater accessibility to membranous intracellular organelles and cytoplasmic locations promote the accumulation of RNAs in sEVs. Since most RNAs are relocated to specific cellular compartments in association with RNA-binding proteins (RBPs) and 25% of sEV proteins have been identified as RBPs, it is rational to assume that RBPs are important in transferring RNAs into sEVs (35, 36). For example, Beltri et al. reported that a four nucleotide motif (GGAG) could bind to sumoylated heterogeneous ribonucleoprotein A2B1 (hnRNPA2B1), thus delivering miRNAs into sEVs derived from human T cells (37). HnRNPA2B1 could also deliver unspliced HIV genomic RNA into sEVs *via* the interaction with several sequences (A2RE and nucleotides 557-663) (38, 39). Besides, miRNAs with 3′-end uridylation appeared to be directed into sEVs but 3′-end adenylated isoforms were more likely to be confined within the cells, indicating that post-transcriptional modification plays a role in the RNA sorting system (40, 41). Subsequently, RNA secondary configuration and unique motifs (42, 43), the interaction with membrane lipids (43) and innumerable RBPs, such as AG02 (44), major vault protein (MVP) (45), YBX1 (46, 47) and lupus La protein (48), have also been implicated in RNA packaging into sEVs. In summary, there are multiple mechanisms of cargo sorting and ILVs formation and it is still obscure whether the sequestering and sorting of specific molecules requires different pathways or how these pathways regulate various ILV subpopulations even within one MVB.

The components of sEVs indicate their cellular origin and potential biological functions. As oncologists, we have a particular interest in identifying sEV-related oncogenic factors (49–52). Significant efforts have been made to characterize the oncogenic alterations in sEVs and inhibit tumor-specific sEV pathways as a new class of anticancer therapies. Here, we briefly discuss how the malignant transformation of parent cells affects sEV components to promote cancer progression and described sEV as cancer biomarkers. For instance, upregulation of oncogenes can increase the levels of sEV oncoproteins, such as EGFR variant III and HRS (53, 54). Additionally, researchers have reported specific collections of sEV proteins associated with different donor cells. For example, Hurwitz et al. reported that nine different cancer types had only 213 sEV proteins in common through proteomic analysis of sEVs from 60 cancer cell lines provided by the National Cancer Institute (NCI-60). Most of the 6,071 proteins identified were unique for each cancer type, suggesting that sEV protein enrichment analysis could provide insight into the cells of origin (55). In line with these findings, p53 loss and oncogenic aberrations in EGFR in human bronchial epithelial cells (HBECs) leads to sEV protein patterns that are distinct from those in non-malignant HBECs (52).

Nucleic acids and lipid components can also be altered by oncogenic mutations (56, 57). In patients with non-small-cell lung cancer (NSCLC), the levels of let-7f and miR-30e-3p in circulating sEVs are positively correlated with disease severity (58). Llorente et al. showed that, compared with parental cells, sEVs from prostate cancer cells had significant enrichment of distinct lipids and a higher lipid-to-protein ratio, indicating that the lipid profile of sEVs could provide further information about sEV biogenesis (59).

Numerous randomized clinical trials have revealed different clinical outcomes in patients with the same cancer after treatment with different therapeutic regimens, raising the possibility that different treatments or stress factors in tumor cells can alter sEV cargo patterns and downstream signaling pathways. Harmati et al. obtained B16F1 cell-derived sEVs released under heat, oxidative, or cytostatic stress and observed unique miRNA and protein patterns in each sEV group (60). Besides, each sEV group demonstrated distinct oncogenic functions; for instance, doxorubicin-elicited sEVs enhanced melanoma cell migration, and oxidative stress-elicited sEVs promoted Ki-67 upregulation in mesenchymal stem cells (60). These results suggest that we may be able to predict therapeutic outcomes and design more effective personalized cancer treatment plans based on the analysis of sEVs from the patients’ tumor tissue, organoid models, or xenograft models. Using these models, we could precisely mimic the complex tumor microenvironments and obtain reliable information about the disease.

## Small Extracellular Vesicles and Cancer Development

Recently, the importance of sEVs in intercellular communication has attracted increasing attention, especially in the context of tumorigenesis and metastasis. The bilayer lipid membranes of sEVs protect their cargo, enabling the transfer of signaling molecules from sEVs to the nearby cells or the distant sites *via* circulatory and lymphatic systems (61–64). It has become evident that sEVs from cancer cells can promote tumor progression and metastasis through multiple pathways (65–68). For instance, breast cancer-derived sEVs promoted oncogenic transformation in non-malignant epithelial cells (65, 69, 70), neoangiogenesis (71–73), cancer cell invasion, metastasis (74), chemoresistance (75, 76), and immune suppression (77, 78). Recently, Gao et al. reported that cancer-associated fibroblasts (CAFs) promoted tamoxifen resistance in breast cancer by sending miR-22 to silence ERα and PTEN expression in recipient cancer cells, suggesting the engagement of tumor stroma-derived sEVs in oncogenesis (79).

Additionally, sEVs may serve as “waste disposals” to eliminate unwanted cellular components (8, 9). Recent studies have identified the crosstalk between lysosomal degradation, autophagy and sEV biogenesis (80). As a traditional proton pump V-ATPase inhibitor, bafilomycin A1 could increase the pH of lysosomes and interfere with the trafficking between lysosomes and other intracellular compartments, especially MVBs and autophagosomes, thus enhancing sEV secretion in various cell types (81, 82). Some researchers reported that bafilomycin A1 could remarkably reduce the tumor load in hepatocellular carcinoma(HCC) xenograft mice and confirmed its potential as antitumor medicine (83). However, this conclusion is challenged by other experiments. Guo et al. discovered that the autophagy-related protein 5 (ATG5) could improve sEV secretion by dissociating V1V0-ATPase that acidifies MVBs and lysosomes, similar to the mechanism that bafilomycin A1 promoted sEV secretion; the increased sEV secretion could accelerate tumor migration in breast cancer mice models (84). These conflicting results may be due to the relatively small sample size of animal experiments, different cell types, and more importantly, the intricate relationship between sEV secretion and autophagy, warranting extensive investigation to illuminate the underlying mechanism.

Another interesting study showed that bafilomycin A1 could rescue the sEV secretion from human T cells, which was impaired by the IFN-1 induced TSG101(a component of ESCRT complex) ISGylation (85). In a ubiquitin-like fashion, interferon-stimulated gene 15 (ISG15) is covalently linked to target proteins, a process called ISGylation. Some researchers reported that downregulation of ISG15 increased the camptothecin resistance in breast cancer, while another study showed that high ISG15 expression in breast cancer indicated radiation resistance and poor prognosis (86, 87). Therefore, bafilomycin A1 might serve as a powerful tool to help us understand the double-edged sword role ISGylation plays in oncogenesis with a mechanism involving membrane vesicle trafficking.

## Small Extracellular Vesicle Biomarkers

### Protein Biomarkers for Cancer Diagnosis

ExoCarta is a manually curated database of sEVs proteins, RNAs and lipids, providing imperative information for sEV research. As of January 21, 2021, the number of recorded protein (9,769) has far exceeded that of RNAs (3,408) and lipids (1,116), indicating extensive studies on sEV proteins (88). Therefore, it is safe to suppose that sEV proteins could function as biomarkers for sEVs-related biological events. Several proteins, such as CD9, CD63, and CD81, are enriched on most sEVs and recognized as markers to verify the presence of sEVs in heterogeneous populations of EVs (89). Further research showed that some unique sEV proteins were associated with the existence of tumor cells, thus facilitating the early cancer detection and prognosis prediction (**Table 1**).

**Table 1:** sEV protein markers in multiple cancers.

Tumor types	Human sample	Isolation methods	Signature proteins	Possible application	Ref.
Lung cancer	Blood	Ultracentrifugation	LG3BP and PIGR	Diagnosis	(90)
	Saliva	Ultracentrifugation	BPIFA1, CRNN, MUC5B, and IQGAP	Detection	(91)
	Urine	Ultracentrifugation	LRG1	Diagnosis	(92)
Breast cancer	Plasma	Ultracentrifugation	144 Phosphoproteins	Detection	(93)
	Serum	Ultracentrifugation	Survivin and Survivin-ΔEx3	Prognosis	(94)
	Plasma	Ultracentrifugation	FAK	Diagnosis and prognosis	(95)
Pancreatic cancer	Blood	Ultracentrifugation	Glypican-1	Diagnosis	(96)
	Plasma	Ultracentrifugation	MIF	Prognosis	(66)
Colorectal cancer	Plasma	ExoCap™ kit	GPC1	Diagnosis	(97)
	Blood	Ultracentrifugation	CD147	Detection and diagnosis	(98)
Ovarian cancer	Ascitic fluid	Ultracentrifugation	TGM2, U2AF1, U2AF2, and HNRHPU	Diagnosis	(99)
Glioma	Cerebrospinal fluid	Ultracentrifugation	IL13QD	Detection	(100)
Cholangiocarcinoma	Blood	Ultracentrifugation	VNN1, CRP, FIBG, IGHA1, and A1AG1	Diagnosis	(90)
Melanoma	Plasma	Ultracentrifugation	MIA and S100B	Prognosis and diagnosis	(101)
Prostate cancer	Urine	Ultracentrifugation	PCA3	Diagnosis and monitoring	(102)

The application of sEVs as liquid biopsy samples has gained substantial attention (**Figure 2**). Although blood is the primary sample used for liquid biopsy, saliva is a promising alternative approach to detect early-stage oral cancer since obtaining saliva is less invasive and closer to malignant lesions than phlebotomy. For instance, increased expression of alpha-2-macroglobulin, haptoglobin, and mucin-5B on oral cancer-derived sEVs could serve as biomarkers for oral cancer diagnosis (103). Saliva biopsies are also becoming increasingly common for head and neck cancer diagnosis, in addition to the detection of other solid tumors, such as breast cancer (104) and pancreatic cancer (105, 106). Urinary sEV protein analysis also identified several markers associated with pancreatic cancer and has emerged as another noninvasive method to identify biomarkers for cancer diagnosis (107).

**Figure 2:** Clinical applications of sEVs TAA, tumor-associated antigens; DAMPs, damage-associated molecular patterns; NKG2D, Natural Killer Group 2D receptor ligands.

Some surface proteins can guide the cellular tropism of sEVs, leading to organotypic metastasis. For instance, breast cancer-derived sEVs coated with integrin α6β4 and α6β1 were more likely to be uptaken by pulmonary fibroblasts and epithelium, establishing a premetastatic niche in the lungs (74). Several surface proteins from melanoma-derived sEVs, such as very late antigen 4 (VLA-4) and tyrosinase-related protein-2 (TYRP2), were also shown to recruit bone marrow progenitor cells to premetastatic niches *via* the MET signaling pathway, promoting bone metastasis and outgrowth (67, 108). Compared with without liver metastasis and healthy control subjects, stage 1 pancreatic ductal adenocarcinoma (PDAC) patients who later developed liver metastasis had remarkably higher levels of migration inhibitory factor (MIF) in their circulating sEVs (66). Depletion of MIF in PDAC-derived sEVs strongly inhibited the formation of fibrotic microenvironment created by Kuffer cells, thereby reducing premetastatic niche in preclinical mice models (66). These unique surface proteins could potentially be used to predict metastatic sites.

However, to which extend a single sEV protein marker can serve as a diagnostic and predictive biomarker in cancer is still under debate. Glypican 1 (GPC1) levels on pancreatic cancer-derived sEVs indicated cancer burden in patients before and after surgery, exhibiting significant diagnostic and predictive potentials (96, 109). In contrast, other studies have failed to confirm the diagnostic value of GPC1 alone in pancreatic cancer (110), highlighting the need for the combination of GPC1 with other biomarkers to increase diagnosis accuracy (111, 112). These studies emphasize that we could not sensitively detect early-stage cancerous lesions with a single protein biomarker, probably owing to the high heterogeneity of tumors.

### Protein Biomarkers of Immunotherapy Response

Certain sEV proteins have been shown to modulate the tumor immune microenvironment through various mechanisms. Notably, the melanoma-derived sEV cargo proteins S100A8 and S100A9 downregulated the expression of the costimulatory marker CD83 in dendritic cells (DCs), thereby inhibiting DC maturation and cytokine production, as well as establishing a premetastatic niche (113). In melanoma mouse models, sEVs containing high PD-L1 levels have been shown to bind PD-1 receptors on T cells, exacerbating T cell exhaustion; pembrolizumab administration diminished this immunosuppression (77, 78). Therefore, further investigations of circulating PD-L1^+^ EVs are required to identify the mechanisms underlying anti-PD-L1 therapy failure and determine the ability of PD-L1^+^ sEVs to predict clinical outcomes of anti-PD-L1 treatment (**Figure 2**).

Intriguingly, blockade of PD-L1^+^ sEVs reinforced systemic antitumor responses in mouse models of prostate cancer (78), underpinning these cancer-promoting sEVs as a promising therapeutic target. Several studies have demonstrated that PD-L1 on sEVs acts as a decoy inhibiting immune responses in draining lymph nodes (78, 114, 115). Furthermore, increased levels of serum PD-L1^+^ sEVs predicted poor prognosis in patients with head and neck cancer (116). Although these data suggest serum PD-L1^+^ as a promising predictor of immunotherapy response and that targeting tumor-associated sEVs may augment the antitumor effects of immunotherapy, the underlying mechanisms remain unclear. In addition to immune checkpoints, tumor-infiltrating lymphocytes and innate immune cells are also crucial for the success of immunotherapy (117, 118). However, future studies are required to confirm the ability of circulating PD-L1^+^ sEVs to predict response to anti-PD-L1 therapy.

sEVs also play a critical role in innate immune responses. Pancreatic cancer-derived sEVs were found to express tumor-associated antigens (TAA)(Fig.2) and bind to circulating autoantibodies, thereby inhibiting complement-mediated cancer cell lysis (119). Furthermore, gastric cancer cell-derived sEVs were enriched in high mobility group box-1 (HMGB1) and activated tumor-promoting neutrophils *via* the TLR4/NF-κB signaling pathway (120). However, a recent study has shown that sEVs released by breast cancer cells with higher expressing of NFAT3 could inhibit cancer cell invasion; the underlying mechanisms are under extensive investigation (121). It is widely accepted that tumor-associated sEVs are key modulators of immune responses, exerting anti-inflammatory or pro-inflammatory effects. Therefore, sEVs can be used as robust biomarkers to predict cancer prognosis and response to immunotherapy (122).

### Nucleic Acid Biomarkers

In addition to protein sEV cargoes, nucleic acids contained in sEVs have also emerged as promising biomarkers. Nucleic acid components include DNA, coding mRNA, and non-coding RNA (ncRNA) molecules (13, 123). Double-stranded (ds) mitochondrial and genomic DNA molecules have been detected in serum sEVs from cancer patients (124, 125). Importantly, sEV dsDNA reflected driver mutations in patients with pancreatic cancer (50, 126, 127). In addition to shared genetic mutation patterns, sEV DNA and genomic DNA have similar nucleic acid modifications. Thakur et al. have identified shared methylation patterns between sEVs DNA and chromosomal DNA from parental cells, suggesting that sEV DNA methylation analysis might have strong clinical implications (126).

Ten HCC-related mRNAs in sEVs were identified by EV Click Chip analysis and these mRNAs could be used to accurately detect early-stage HCC (128). A scoring system based on these mRNAs was superior in distinguishing HCC patients from liver cirrhosis patients. Compared with traditional serum AFP tests, this system provided a higher area under the curve (AUC) of 0.69 versus 0.93, 0.68 versus 0.91, and 0.70 versus 0.92, according to BCLC stage 0-A, Milan criteria, and UNOS DS criteria respectively (128). These data provide strong evidence of sEV mRNA utilization for early-stage cancer detection.

ncRNAs, such as microRNAs (miRNAs), circular RNAs, and long ncRNAs (lncRNAs), are also abundant in sEVs (36, 129). The levels of certain miRNAs have been associated with cancer development and progression (130–132). Several studies have shown that, in HCC patients, high levels of miR-92a-3p in circulating HCC-derived sEVs were associated with HCC cell proliferation and poor overall survival (130, 133, 134). In multiple myeloma-derived sEVs, let-7b, and miR-18a levels accurately stratified patients according to survival outcomes (132). Although one or two specific miRNAs could strongly predict cancer prognosis, a recent study has shown that using a miRNA signature improves the sensitivity and specificity of sEVs as biomarkers (135–137). A miRNA cluster from breast cancer-derived circulating sEVs has been confirmed as a predictor for bone metastasis and is currently under investigation as a new therapeutic target (138).

ncRNAs from sEVs are also promising clinical biomarkers. In cholangiocarcinoma, several lncRNAs (139) and circular RNAs (140, 141) from circulating sEVs have been correlated with metastasis and have been proposed as cancer biomarkers (142). An ongoing clinical trial is investigating the ability of a group of serum lncRNAs to detect early-stage lung tumors to improve clinical outcomes (143).

An obstacle in the discovery of liquid cancer biomarkers is the low yield of sEV isolation methods, which are not yet suitable for clinical practice. Genetic engineering of donor cells and manipulating the cell culture medium have been employed to scale up the isolation of sEVs (144). Furthermore, many techniques have been established to purify sEVs based on their unique physicochemical and biochemical properties (145, 146). Particularly, sEV isolation by size-exclusion separation chromatography can significantly reduce the sEV damage and protect sEV nucleic acids and other cargoes (145).

### Lipid Biomarkers

Compared with sEV proteins and nucleic acids, sEV lipids have been studied less as cancer biomarkers, possibly due to the limited diversity in sEV lipids and the limitations of lipid analysis techniques. In 2003, distinct lipid patterns were identified in sEVs from human B cells. The accumulation of certain lipids and a relatively higher lipid-to-protein ratio were also validated in sEVs secreted by colorectal cancer cells and prostate cancer cells (**Figure 2**) (59, 147). Recent studies evaluated the lipidomic profiles of cancer-derived sEVs. Cheng et al. have demonstrated that sEVs from human ovarian cancer cells SKOV-3 had higher amounts of cholesterol esters and zymosterol species than sEVs derived from a different human ovarian epithelial cancer cell line (HOSEPiC), indicating that the lipid profile of sEVs could indicate the origin of sEVs (148). However, considering that these cholesterol esters assemble dynamically into lipid rafts and are rapidly exchanged between neighboring cells, future studies are warranted to determine the feasibility and sensitivity of using cholesterol esters as cancer biomarkers.

## Modified Small Extracellular Vesicles for Cancer Therapy

In the past decade, we have witnessed the exponential growth of sEVs modification strategies. These strategies could be classified into two types according to the source of parental cells: altering sEVs from unmodified parental cells and harvesting sEVs from well-modified parental cells (**Figure 3**).

**Figure 3:** Modified sEV as anticancer therapies.

### Alteration of Small Extracellular Vesicles From Unmodified Donor Cells

#### Increasing Targeting Ability of Small Extracellular Vesicles

Numerous efforts have been made to increase the targeting ability of modified sEVs. Aminoethylanisamide-polyethylene glycol (AA-PEG) vector moiety targeting the sigma receptor on cancer cells was integrated into sEVs from macrophages *via* crosslinkers (149) (**Figure 2**). Compared with unmodified parental sEVs, modified sEVs accumulated in cancer cells and prolonged overall survival in mice (149). Tian et al. established an efficient and rapid method to add integrin αvβ3 targeting peptides [c(RGDyK)] onto the sEVs *via* crosslinkers, considering the high expression of integrin αvβ3 on the surface of reactive vascular endothelial cells (150) (**Figure 3**). Although this technology was initially employed in cerebral ischemia models, it can be adapted for anti-angiogenesis therapy in cancer models, given the role of integrin αvβ3 in promoting tumor angiogenesis (151). Modified nucleic acids could also be used for targeted delivery. Pi et al. developed an innovative method to anchor arrow-shaped RNA nanoparticles, known as aptamers, on the surface of sEVs, which carried therapeutic siRNA and miRNA (152). These aptamers could be stably attached to the external surface of the membrane due to their unique configuration and the cholesterols added to their tails (152) (**Figure 3**). The aptamers specifically recognized surface cancer markers, such as EGFR in breast cancer and PSMA in prostate cancer, thus guiding the sEVs to cancer cells (152).

Compared with EVs from genetically engineered donor cells, surface-modified purified sEVs provides more options in terms of conjugated ligands. However, how to protect sEV structure and cargoes from acidic environments and high-speed centrifugation in the modification process are critical challenges that need to be addressed.

#### Loading Isolated Small Extracellular Vesicles With Functional Molecules

Compared with liposomes, carbon nanoparticles, and other artificial drug delivery systems, autologous sEVs are less toxic and immunogenic (153, 154). sEVs can also target tumor cells and immune cells with a higher specificity than liposomes and are ideal drug delivery vehicles (155, 156). Numerous efforts have been made to engineer isolated sEVs and donor cells (**Figure 3**). Some commercial kits have been available for loading nucleic acids into sEVs (64). The techniques used to load sEVs with various cargo include free-thaw cycles to fuse sEVs and liposomes, sonication, extrusion, permeabilization with saponin, and electroporation (157–159). Electroporation is commonly used to transfer small interfering RNAs (siRNAs) and other cytotoxic agents into sEVs (160–164). Particularly, mesenchymal stromal cell-derived sEVs loaded with siRNA or other oligonucleotides specific for oncogenic Kras^G12D^ strongly inhibited Kras^G12D^ expression in pancreatic ductal cancer cells and inhibited orthotopic tumor growth (162). Importantly, sEVs loaded with Kras^G12D^-targeting siRNA significantly suppressed pancreatic cancer growth in mice (162). The strong antitumor effects of these modified sEVs were attributed to their high CD47 levels, which protected sEVs from macrophage-mediated elimination (162). Recently, Faruqu et al. used electroporation to transfer siRNAs into sEVs from human embryonic kidney cells (HEK-293 cells); these modified sEVs were internalized by pancreatic cancer cells with high efficiency, providing a standard procedure for making siRNA-containing sEVs *via* electroporation (164) (**Figure 3**). Although sEV loading by electroporation may cause less damage than the genetic modification of donor cells, RNA precipitation and altered biochemical and physiochemical features of the membrane during electroporation are critical challenges that need to be addressed (165).

### Therapeutic Small Extracellular Vesicles From Modified Donor Cells

#### Enhancing the Targeting Ability of Small Extracellular Vesicles

Although the ability of sEVs to target different cell types has been well demonstrated, their targeting ability as a drug delivery system can be further enhanced by introducing targeting molecules into the donor cells, which release the targeting ligand-enriched sEVs. The neuron-targeting peptide RVG has been successfully conjugated with Lamp2b, a transmembrane protein abundantly found on the surface of sEVs (161, 166). This reconstructed protein enabled the delivery of therapeutic siRNA-packaged sEVs to neurons, maximizing their safety and efficacy (161). Although this method was primarily tested in mouse models of neurodegenerative diseases, it provided an optimized method to improve the targeting ability of sEVs. Recently, HEK293T cell-derived sEVs with Lamp2b-anti-HER2 affibody fusion protein were shown to selectively bind HER2-expressing colon cancer cells, delivering 5-fluorouracil and miRNA inhibitors to tumor cells and suppressing tumor growth (**Figure 3**) (167).

Significant progress has also been made in combining various nanoparticles and sEVs *via* chemical modification of donor cell membranes, providing a novel method to generate therapeutic sEVs. For instance, nanobodies attached to the sEV surface *via* a glycosylphosphatidylinositol (GPI) linker can recognize different therapeutic targets, such as EGFR expressed on tumor cells (**Figure 3**) (168, 169).

#### Chemotherapeutics Cargo

Modification of donor cells is another strategy to load anticancer agents into sEVs and improve the targeting ability of sEVs. An early study showed that paclitaxel-treated donor cells secreted paclitaxel-containing sEVs, which significantly inhibited the proliferation of pancreatic cancer cells *in vitro* (170). Guo et al. designed a novel system to generate methotrexate (MTX)-loaded EVs from UVB-irritated donor cells treated with MTX previously (**Figure 3**) (171). These EVs (30–930 nm in diameter) remarkably increased the overall survival of mice with malignant pleural effusion and decreased pleural effusion in a small group of patients with late-stage lung cancer (171). These preliminary findings open a new avenue for the production of therapeutic EVs by manipulating donor cells. However, the clinical implementation of this method is hindered by several factors. Importantly, a balance between achieving an ideal loading efficacy and minimizing cytotoxicity caused by co-incubation with chemotherapy drugs is required. The stability of the pharmaceutics in the cytoplasm is another key concern, given that some commonly used drugs (e.g., cisplatin and paclitaxel) can be inactivated by intracellular enzymes (170, 172, 173). Indeed, isolated sEVs, rather than intact donor cells, have been regarded as more suitable carriers to transport chemotherapeutics because of the limitations of current techniques and platforms.

#### Protein Cargoes

##### Single Soluble Proteins

Transfecting donor cells with vectors carrying genes of interest is a possible method to generate sEVs enriched in specific proteins. Previous studies have reported the successful generation of sEVs carrying 5-fluorocytosine-activating enzymes by transfecting 293T cells; co-administration of these sEVs with 5- fluorocytosine significantly inhibited the proliferation of glioma cells (**Figure 3**) (174, 175). The feasibility of this method has been validated by a study showing that caspase-1-containing sEVs released from transfected 293T cells inhibited the growth of schwannoma cells without causing significant neurotoxicity (176). However, this sEV generation approach has been used less than the production of siRNA/miRNA-enriched sEVs. One of the challenges in producing soluble protein-enriched sEVs is the cytotoxicity to parental cells caused by the overexpression of these proteins, which significantly reduces sEVs production yield and alters sEV composition (174). Another obstacle is the complexity of the protein sorting and trafficking system involved in sEV biogenesis. This system randomly delivers target proteins into sEVs, hindering the reproducibility of the method (174, 177). Therefore, other approaches have been established to specifically transport target proteins into sEVs, including conjugation of the target protein with sEVs-associated proteins and ubiquitination of target proteins.

##### Recombinant Proteins

Enhancing the expression of target proteins and exogenous leader peptide complexes in donor cells has emerged as a promising method to generate sEVs. Viral envelope proteins are an ideal source of leader peptides. The mechanisms underlying viral recognition of target cells and viral spread *via* cellular vesicles have been extensively studied for decades, and several links between viral proteins and sEV biogenesis have been identified (178, 179). Viral proteins can be delivered to sEVs by using endosomal sorting complexes required for transport (ESCRT). CD8 ectodomain-Env chimeric protein was loaded to K562 cell-derived sEVs by the interaction of the Env protein of the bovine leukemia virus with ESCRT (180). A mutated HIV-Nef protein, also known as Nef^Muf^, was transported to sEVs without causing significant damage, indicating its potential to lead target molecules to sEVs (181–183). Manfredi et al. designed a Nef^Muf^/E7 DNA carrier to incorporate Nef^Muf^-HPV E7 fusion protein into 293T cell-derived sEVs (184). The HPV E7 protein conjugated to the C-terminal of Nef^Muf^ accumulated in the sEVs; these sEVs remained intact and activated anti-E7 CD8^+^ T cells, inhibiting TC-1 tumor cell proliferation in mice (**Figure 3**) (184). Vesicular stomatitis virus glycoprotein (VSVG) among other viral proteins, has also been used as leader peptides to target fusion proteins into sEVs (185). Therefore, viral leader peptides may provide a novel avenue to produce therapeutic sEVs.

Interestingly, some intracellular signal tags have been demonstrated to facilitate the targeted delivery of modified molecules to sEVs. Cheng et al. reported that recombinant proteins with C-terminal ubiquitination were ten times more likely to be loaded into HEK 293 cell-derived sEVs than unmodified isoforms (186); sEVs carrying ubiquitin (Ub)-tagged proteins boosted T cell responses (**Figure 3**) (186). Additionally, monoubiquitinated syntaxin 3 (Stx3) was rapidly internalized from the basolateral plasma membrane and was secreted apically into sEVs along with Stx3-binding partners (187). However, mutated forms of Stx3 that cannot be ubiquitinated could not be loaded into sEVs and reduced the shedding of human cytomegalovirus (HCMV) from infected cells, highlighting this to be a promising approach to produce customized sEVs (187). Besides, some plasma membrane anchors, such as N-terminal myristoylation and palmitoylation, selectively guided fusion proteins to sEVs (188). Sterzenbach et al. labeled Cre recombinase with WW tag, a signal peptide recognized by NDFIP1 involved in ESCRT system assembly. The modified Cre recombinase was ubiquitinated and loaded into sEVs (189). Interestingly, the recipient cells underwent Cre-mediated genomic editing after sEV internalization, opening a new avenue for reversing oncogenic mutations in tumor cells (**Figure 3**) (189).

However, one problem of using reconstructed proteins is the fragility of signal peptides during sEV biogenesis (166). Besides, whether these cargo modifications work independently of the ESCRT machinery is still under debate. Studies have shown that ubiquitinated MHCII β-chain levels were withdrawn from the cell surface and accumulated into secretory sEVs (190, 191). In contrast, Gauvreau et al. argued that MHCII molecules are loaded into sEVs *via* a ubiquitin-independent pathway (192). Additionally, it remains unclear whether these tags, especially ubiquitin, induce the degradation of fusion proteins by proteasomes and alter the therapeutic effects of sEVs.

Another possible method to generate therapeutic ligand-enriched sEVs is the conjugation of target proteins with constitutive sEV proteins, especially transmembrane proteins and peptides. These hybrid proteins have successfully been delivered to sEVs and the antitumor effects of these sEVs are under investigation (193) (**Table 2**). For example, CD9 is abundantly found on the sEV surface. Yim et al. developed an optically controlled delivery system by using the interaction between cargo-photoreceptor cryptochrome 2 (CRY2) soluble protein and CIBN-CD9 membrane complex. Under blue light, the interaction between CIBN and CRY2 subunits attaches the cargo protein to the intraluminal site of the sEV membrane, and the cargo can be released into the intraluminal space in the absence of blue light (**Figure 3**) (205). Moreover, sEVs from genetically engineered immune cells, a widely used immunotherapy, can deliver specific proteins to desired organs and cells. Compared with chimeric antigen receptor (CAR)-T cells, sEVs from CAR-T cells caused less severe cytokine release syndrome and comparable antitumor effects in mouse models (206). Moreover, CAR-T cell-derived sEVs with minimal PD-1 expression are less immunosuppressive than CAR-T cells, which express higher levels of PD-1 (206). Therefore, more research is needed to validate these promising preclinical findings and confirm the therapeutic effects of CAR sEVs in patients. Additionally, the ability of CAR sEVs to improve the safety and antitumor efficacy of CAR-T cell therapy merit further investigation.

**Table 2:** Proteins or peptides providing potential modification targets to load therapeutic agents.

Proteins or peptides	Characteristics	reference
CD63, CD9, CD81	Tetraspanin	(194–196)
MHC	Membrane-anchored	(197)
SCAMPs	Secretory carrier-associated membrane protein	(193)
EGF VIII	Transmembrane glycoprotein	(198)
LAMP2B, LAMP1	Lysosome-associated membrane glycoprotein 2, lysosome-associated membrane glycoprotein 1	(199, 200)
PDGFR TM domain	Cell surface tyrosine kinase receptor	(201)
VSVG	Vesicular stomatitis virus glycoprotein	(185)
HSP90, HSP70, HSP50	Heat shock protein	(202, 203)
WW tag	Recognized by the L-domain-containing protein Ndfip1, resulting in ubiquitination and loading into sEVs	(189)
ALIX-1	Cytosolic protein that associates with MVB by interacting with ESCRT-III subunit SNF7	(204)

#### Nucleic Acid Cargo

Due to their natural characteristics, such as low homing in the liver and better penetration across the blood-brain barrier, sEVs have been utilized as reliable bio-shuttles for gene therapy, especially delivering brittle nucleic acid agents to target cells (207). Since miRNA and siRNA are the most favorable tools to regulate genomic expression, many efforts have been made to produce sEVs containing miRNAs as therapeutic agents by transfecting donor cells with DNA vectors (208). sEVs from mesenchymal stem cells carrying miR-122 expression plasmids delivered enormous amounts of miRNAs to liver cancer cells, sensitizing xenograft tumors to sorafenib (209). Abels et al. isolated miR-21-enriched sEVs from transfected glioma cells; these sEVs were internalized by microglia and suppressed the expression of specific mRNA targets (210). Although cell transfection is a simple and feasible approach to generate siRNA-enriched sEVs, cytoplasmic siRNA instability and miRNA-mediated cytotoxicity in donor cells are challenges that remain to be addressed.

## Other Therapeutic Applications of Small Extracellular Vesicles In Cancer

### Depletion of Cancer Cell-Derived Small Extracellular Vesicles

Given that cancer cell-derived sEVs promote cancer progression and metastasis, the depletion of circulating oncogenic sEVs has been proposed as a method to suppress cancer progression (172, 211). In xenograft mouse models of human breast cancer, administration of anti-CD9 and anti-CD63 antibodies suppressed the spread of cancer cells to lymph nodes, lungs, and the thoracic cavity by targeting cancer-derived sEVs carrying CD9 and CD63 (212). Subsequent studies have demonstrated the preferential internalization of antibody-tagged sEVs by macrophages, suggesting that blocking specific surface protein biomarkers on sEVs could be a promising anticancer strategy (212).

Aptamer-modified nanoparticles were employed to transport circulating lung cancer-derived sEVs from the circulation to the intestinal tract; these agents inhibited sEV-induced metastasis in mice. Notably, EGFR-targeting aptamers were attached to positively charged mesoporous silica nanoparticles, and when they were injected intravenously, they recognized circulating EGFR^+^ sEVs. sEVs-nanoparticle complexes were uptaken by Kuffer cells and secreted into the bile; their elimination from the circulation suppressed cancer cell metastasis (211). Hence, selective depletion of circulating oncogenic sEVs can improve therapeutic outcomes in cancer patients and imply various potential clinical applications.

Chemotherapy and radiotherapy can cause the accumulation of DNA fragments in the cytoplasm of cancer cells and some DNA pieces are disposed of into sEVs (213–215). As sEVs could remove damage-associated molecular patterns (DAMPs) from source cells to maintain intracellular homeostasis, inhibiting sEVs secretion can increase DAMPs levels in the cytoplasm, triggering cancer cell apoptosis (214). Cannabidiol, ketotifen, and simvastatin can block sEV biogenesis and release from cancer cells and monocytes through various mechanisms, which amongst others are linked to mitochondrial dysfunction and calcium dysregulation, thereby reversing chemotherapy resistance and magnifying antitumor immune responses (216–219). Interestingly, these inhibitors target different steps of sEV biogenesis and secretion; thus, combination therapies could synergistically inhibit sEV secretion.

### Small Extracellular Vesicles as Vaccines

Numerous research has focused on developing cancer vaccines to augment antitumor immunity. In April 2001, the US Food and Drug Administration (FDA) approved Provenge^®^ (sipuleucel-T) as the first cancer vaccine to treat metastatic, hormone-resistant prostate cancer (220, 221). Unlike traditional prophylactic vaccines against infectious diseases, this anticancer vaccine primes DCs with prostate cancer-associated antigens *in vitro*, and the activated DCs are then re-infused into patients (222). In a phase III trial, sipuleucel-T significantly prolonged the overall survival of 127 patients with metastatic prostate cancer survival without causing significant toxicity (223). However, not all clinical trials of sipuleucel-T showed encouraging results (224), raising the need for further investigation of the clinical efficacy of sipuleucel-T. The inconsistent clinical outcomes may be due to the variable sensitivity of DCs to immunosuppressive molecules, and the cost of priming and storing autologous DCs is very high. Therefore, we wonder whether cell-free vaccines, such as sEV-based vaccines, could facilitate antitumor immunity. Cancer cell-derived sEVs could carry numerous tumor-associated neoantigens, MHC class I molecules and HSP70, which are recognized as the stimulus for the immune response against cancer (225, 226). Rao et al. showed that HCC-derived sEVs could carry several HCC-associated antigens and trigger a stronger tumor suppression than cell lysates in murine HCC models (227). Biopsy showed improved HCC tumor microenvironments by sEVs, with increased T lymphocyte infiltration, elevated IFN-γ and decreased interleukin-10 expression, indicating sEV cancer vaccines as competent immune modulators (227).

DAMPs involved pathways have also been reported in the application of sEV cancer vaccines. Due to the hypoxia, malnutrition and cytotoxic agents in tumor microenvironments, misfolded proteins accumulate in cancer cells and trigger endoplasmic reticulum (ER) stress (228). ER stress could promote MVB formation and the release of the DAMPs-rich sEVs, which could inhibit tumor progression *via* an inflammatory response (229, 230). DNA fragments resulted from chemotherapy are a well-known example of DAMPs. For instance, chromosomal DNA-rich sEVs from cancer cells treated with topotecan activated DCs *via* the cGAS-STING signaling pathway, thereby inducing cancer cell apoptosis and inhibiting tumor progression (213, 231, 232). Given that these sEVs may promote antitumor immunity, careful selection of DNA-containing sEVs subpopulations is critical.

Furthermore, sEVs from irradiated cancer cells could inhibit the growth of nearby nonirradiated cells, a phenomenon known as the radiation-induced bystander effect (RIBE) (233). Numerous sEV contents have been identified to mediate the RIBE, including cytokines, antigens, free radicals, and immune modulators (234, 235). For instance, high levels of miR-1246 have been detected in sEVs from irradiated BEP2D cells, and miR-1246 has been shown to inhibit non-homologous end joining (NHEJ) and the proliferation of unirradiated recipient cells (236). Besides, several studies have shown that adjusting wavelengths and doses of electromagnetic radiation could remarkably alter the number of sEVs produced by mesenchymal tissues and tumor cells *via* several mechanisms, such as the activation of Wnt signaling and enhanced p53 expression (228, 235, 237, 238). These results indicate that not only the contents but the number of sEVs might account for RIBE, which varies with the adaptation of radiotherapy modalities. In a recent study, Wan et al. reported that injecting irradiated lung cancer cell-derived EVs with a mean diameter of approximately 400 nm into the pleural space activated macrophages and significantly prolonged overall survival in a pleural malignancy mouse model (239). Therefore, we wonder if the administration of larger EVs in addition to sEV vaccines could significantly augment the antitumor immunity. These inspiring results have deepened our understanding of RIBE, indicating advanced clinical strategies when managing patients with inoperable cancerous lesions.

Although tumor cell-derived sEVs could perform as potential cell-free vaccines, the culture and expansion of patients’ tumor cells *in vitro* is time-consuming in clinical practice. Malignant effusion, such as ascites from colorectal cancer (CRC) patients, provides an approachable source of adequate tumor cell-derived sEVs. Dai et al. conducted a phase I clinical trial of treating CRC patients with either ascites-derived sEVs alone or the sEVs plus GM-CSF. The combination regimen (sEVs plus GM-CSF) showed remarkable tumor inhibition and confirmed biosafety while administering sEVs alone did not achieve a significant therapeutic effect (240). This study offered a convenient and safe method to harvest autologous sEVs, but the researchers did not compare the clinical outcomes of using GM-CSF alone with the combinatory therapy, requiring more investigation to demonstrate how ascites-derived sEVs enhance antitumor immunity in conjugation with immune-modulatory cytokines (240).

Some immune cells-derived sEVs could also regulate antitumor immunity. DC-derived sEVs (DEVs) carry peptides/MHC complexes, costimulatory molecules, such as CD80 and CD86, and tumor-associated antigens to prime T cells directly *in vitro* (241). However, *in vivo* experiments showed that DEVs were less able to prime naïve T cells *via* direct sEVs-to-T cells interaction (240). Instead, DEVs could be internalized into or fuse with nearby APCs and tumor cells, followed by the antigen presentation on the surface of these recipient cells indirectly (242). Zitvogel et al. reported that cancer cells cocultured with DEVs could more efficiently reactivate previously primed T cells, showing the higher expression of interferon-γ (IFN-γ) (243) Besides, DEVs possess Natural Killer Group 2D receptor ligands (NKG2D-L), which bind to NKG2D on NK cell surface and activate NK cells; the tumor necrosis factor (TNF) in these sEVs could enhance the INF-γ release from NK cells (244). A completed phase II clinical trial conducted in advanced lung cancer patients confirmed the biosafety and activation of NK cells when using DEVs as the maintenance immunotherapy (245). Therefore, DEVs in combination with NK cells for cancer immunotherapy should be considerable.

Cytotoxic T cells (CTLs) are key regulators in antitumor immunity and many methods have been adopted to reactive CTLs in tumor microenvironments. One of the problems when applying these methods is that CTLs can hardly penetrate the dense stromal barriers, which shield cancer cells from the CTL-mediated cytotoxicity. As nano-sized particles with the better penetration across biological barriers, CTL-derived sEVs could efficiently approach the lesions, carry TCR and costimulatory molecules to bind to peptides/MHC complexes and contain cytotoxic enzymes to trigger targeted cell death (246). A recent study reported that with the stimulation of IL-12, high-affinity CTLs could secrete sEVs that activated low-affinity CTLs to produce more granzyme B and IFN-γ (247). However, Xie et al. reported that sEVs from exhausted CD+8 T cells could impair the activity of functional CD+8 T cells and a set of lncRNAs involved in the immunosuppression was identified (246). These paradoxical discoveries allow us to better understand the multiple functions of CTL-derived sEVs under different circumstances and intravital imaging could provide a powerful tool to directly observe the interaction between sEVs vaccines and recipient cells (248). Other source cells for producing therapeutic sEVs have been disclosed, such as NK cells (249), myeloid-derived suppressor cells (MDSCs) (250), tumor-associated macrophages (159), mast cells (251) and neutrophils (252), which shed light on the systemic study of disorganized antitumor immunity.

## Clinical Trials on Therapeutic Small Extracellular Vesicles

As of October 4, 2020, nine clinical trials testing sEVs as potential therapeutics have been registered on ClinicalTrials.gov and Chictr.org.cn (**Table 3**). No sEV-derived therapeutics have been approved by the US FDA or the Chinese National Medical Products Administration (NMPA). The evaluation of the safety and therapeutic efficacy of sEVs remains a significant clinical challenge caused by the lack of understanding of sEV biogenesis and functions. Besides, the pharmacokinetic characteristics of sEVs, such as the rapid clearance through the liver and kidneys, are factors limiting their therapeutic efficacy (201, 253). Notably, nanoparticle drug delivery systems have been approved by the FDA as anticancer agents because of their excellent performance in maximizing the efficacy and minimizing the side effects of chemotherapy (254). Therefore, advancing sEV therapeutics using similar techniques as those used for nanoparticles, such as fusing liposomes with sEV membrane (159) to increase the cellular uptake, improve the performance of sEVs as drug delivery vehicles. Recently, some biotechnology companies have announced plans to start sEV-related clinical trials as early as 2020, providing hope for the clinical application of sEVs (251).

**Table 3:** Registered clinical trials of sVE-related cancer therapies.

Disease	Drug	EV source	Phase, status	Registration number
Metastatic pancreatic cancer	KRAS^c^ G12D siRNA	MSC^d^-derived sEVs	Phase I Recruiting	NCT03608631^a^
Malignant pleural effusion	Methotrexate	Microparticles	N/A Recruiting	NCT04131231^a^
	Methotrexate	Autologous tumor-derived microparticles	Phase II Recruiting	NCT02657460^a^
	Chemotherapeutic drugs	Tumor cell-derived microparticles	Phase II Unknown	NCT01854866^a^
Head and neck cancer	Grape extract	Plant sEVs	Phase I Active, not recruiting	NCT01668849^a^
	Hemopurifier pembrolizumab	Blood-derived sEVs	N/A Not yet recruiting	NCT04453046^a^
Colorectal cancer	Curcumin	Plant sEVs	Phase I Active, not recruiting	NCT01294072^a^
Non-small cell lung cancer	Antigens	Tumor DEV2^e^	Phase II Completed	NCT01159288^a^
Hepatocellular carcinoma	DC-derived vaccine	Hepatic liver cells or other solid tumor cells	Phase I and II Not yet recruiting	ChiCTR1800020076^b^

a The NCT# refers to a registered National Clinical Trial (NCT), which can be found at Clinicaltrials.gov.

b ChiCTR# refers to a registered Chinese Clinical Trial (CHiCT), which can be found at Chictr.org.cn.

c Kirsten Rat Sarcoma (KRAS).

d Mesenchymal Stem Cells (MSC).

e Dendritic Cell-Derived sEVs (DEV).

## Conclusion

In this review, we discuss the role of sEVs in cancer development and the recent advances in using sEVs to diagnose and treat various cancers. Despite significant progress in this field, several important issues remain to be solved. For instance, how to obtain homogenous sEVs subpopulations and distinguish between oncogenic sEVs and antitumor sEVs are significant obstacles in translating these scientific findings into clinical practice. Here, we propose several possible solutions. First, future studies are required to deepen our understanding of sEV biology, such as intraluminal components in different experimental conditions and various downstream events when sEVs are internalized by recipient cells. Second, advanced techniques for large-scale sEV production and purification are in demand. A combinatory approach consisted of immune-magnetic isolation, size-exclusion chromatography, and centrifugation could increase the homogeneity of final products (65, 144, 252, 255, 256). However, this approach could reduce the yield of sEVs due to its multiple steps. Therefore, a balance between obtaining homogenous sEV subpopulations and maximizing sEV yield is required. Establishing a standardized nomenclature system and elucidating the mechanisms underlying sEV biogenesis, release, and interaction with surrounding cells are also required.

Although there are multiple ongoing clinical trials evaluating sEVs as biomarkers for cancer detection and monitoring, only a few clinical trials are investigating the therapeutic effects of modified sEVs; thus, the long-term safety and clinical efficacy of sEVs as therapeutic targets or drug carriers remain unclear. In contrast to using sEVs as drug carriers, inhibiting sEVs release and depleting circulating sEVs are far less studied in preclinical models since sEVs clearance remains a challenge and the available sEV inhibitors cannot selectively inhibit specific sEV subtypes (257). Besides, the biodistribution and safety of sEVs absorption agents is still a major clinical concern (258). Hence, collective efforts are required to address the remaining technical challenges in the development of sEV-based biomarkers and therapies.

## Author Contributions

YG and YQ contributed to the article writing. CW, YS, JM, YH, and JH contributed to the data collection. HJ and KY supervised and revised the article. All authors contributed to the article and approved the submitted version.

## Funding

This study was conducted with the support by the National Natural Science Foundation of China (Grant Nos. 2020BHB021, 81874233, 81874222, and 81672978) and the Key International Cooperation Project of Hubei Province  (82022040).

## Conflict of Interest

The authors declare that the research was conducted in the absence of any commercial or financial relationships that could be construed as a potential conflict of interest.

## Abbreviations

AF4, asymmetric flow field-flow fractionation; ATG5, autophagy-related protein 5; AREG, amphiregulin; CAR-T cells, chimeric antigen receptor T cells; ChiCTR, Chinese Clinical Trials Registry; CRY2, cryptochrome 2; DAMPs, damage-associated molecular patterns; DCs, dendritic cells; DEVs, DC-derived sEVs; EGFR, epidermal growth factor receptor; ESCRT, endosomal sorting complexes required for transport; EVs, extracellular vesicles; GPC1, glypican 1; GPI, glycosylphosphatidylinositol; HBECs, human bronchial epithelial cells; HCC, hepatocellular carcinoma; HCMV, human cytomegalovirus; HEK-293 cells, human embryonic kidney cells; HMGB1, high mobility group box-1; hnRNPA2B1, sumoylated heterogeneous ribonucleoprotein A2B1; HRS, hepatocyte growth factor-regulated tyrosine kinase substrate protein; ISG15, interferon-stimulated gene 15; MDSCs, myeloid-derived suppressor cells; MIF, migration inhibitory factor; MISEV2018, International Society for Extracellular Vesicles in 2018; MTX, methotrexate; MVB, multivesicular body; MVP, major vault protein; NFAT3, nuclear factor of activated T cells 3; NHEJ, non-homologous end-joining; NSCLC, non-small-cell lung cancer; OVA, ovalbumin; PDAC, pancreatic ductal adenocarcinoma; PLP, proteolipid protein; RIBE, radiation-induced bystander effect; sEVs, small extracellular vesicles; SIMPLE, small integral membrane protein of the lysosome/late endosome; Stx3, syntaxin 3; ST6Gal-I, β-galactoside α2,6-sialyltransferase 1; TYRP2, tyrosinase-related protein-2; Ub, ubiquitin; VLA-4, very late antigen 4; VSVG, vesicular stomatitis virus glycoprotein.
